# Research on Small Target Detection Technology Based on the MPH-SSD Algorithm

**DOI:** 10.1155/2022/9654930

**Published:** 2022-11-28

**Authors:** Qingyao Lin, Su Li, Rugang Wang, Yuanyuan Wang, Feng Zhou, Zhaofeng Chen, Naihong Guo

**Affiliations:** ^1^School of Information Technology, Yancheng Institute of Technology, Yancheng 224051, China; ^2^Yancheng Xiongying Precision Machinery Company Limited, Yancheng 224006, China

## Abstract

To address the problems of less semantic information and low measurement accuracy when the SSD (single shot multibox detector) algorithm detects small targets, an MPH-SSD (multiscale pyramid hybrid SSD) algorithm that integrates the attention mechanism and multiscale double pyramid feature enhancement is proposed in this paper. In this algorithm, firstly, the SSD algorithm is used to extract the feature map of small targets, and the shallow feature enhancement module is added to expand the receptive field of the shallow feature layer so as to enrich the semantic information in the feature layer for small targets and improve the expression ability of shallow features. The processed shallow feature layer and deep feature layer are fused at multiple scales, and the semantic information and location information are fused together to obtain a feature map with rich information. Secondly, the cascaded double pyramid structure is used to transfer from the deep layer to the shallow layer so that the context information between different feature layers can be effectively transferred and the feature information can be further strengthened. The hybrid attention mechanism can retain more context information in the network, adaptively adjust the feature map after addition and fusion, and reduce the background interference. The experimental analysis of MPH-SSD algorithm on Pascal VOC and MS COCO datasets shows that the map of this algorithm is 87.7% and 51.1%, respectively. The results show that the MPH-SSD algorithm can make better use of the feature information in the shallow feature layer in the process of small target detection and has better detection performance for small targets.

## 1. Introduction

Target detection technology is a technology to find the target object in the image to be tested with the help of computer vision. This technology can not only realize the target location but also judge the category of the target at the same time. As a key technology in the field of computer vision, small target detection technology has become a hot research topic and thus has a wide range of applications in remote sensing image processing [1, 2] and industry and medicine [3–8].

From the definition of small targets, they are of two types [9], where the first one is to define objects with less than 32 × 32 pixels in the MS COCO dataset as small targets and the second one is to compare the target with the image and define the target as a small target if it accounts for no more than 10% of the image. Because small targets themselves carry less feature information, this is extremely challenging for feature extraction, recognition, and detection [10]. In addition to carrying little information, the small area under the coverage of small targets, single location information, and weak feature representation are all factors that limit the performance of small target detection [11]. The emergence of multiscale feature fusion has provided new ideas to solve these problems, while multiscale fusion strategies have been applied to various image processing tasks, such as super-resolution image processing [12, 13] and semantic segmentation [14, 15].

At present, the mainstream target detection algorithms are mainly divided into one-stage target detection algorithm and two-stage target detection algorithm. Among them, the one-stage target detection algorithm is represented by YOLO series and SSD, which adopts the regression strategy to achieve target detection [16–24], and the two-stage target detection algorithm is represented by classical convolutional neural network algorithms such as R-CNN and fast R-CNN [25–30], and based on the original input image, the candidate region is extracted, and then the image of the candidate region is sent to the convolutional neural network for feature extraction so as to achieve the classification and detection of targets. From the existing research results, the one-stage target detection algorithm does not need to generate a large number of candidate regions, which reduces the detection time and improves the real-time performance of target detection. It has certain advantages in engineering applications and has made good research progress. For example, in 2016, aiming at the problem of different target scales in target detection, researchers such as Liu et al. proposed the SSD (single shot multibox detector) algorithm, which uses feature layers of different scales to detect targets of different scales [31]. However, the algorithm lacks information interaction between shallow and deep information and does not use the feature information between different feature layers, which reduces the detection accuracy of small targets. In order to improve the detection accuracy of small targets, Fu et al. proposed the DSSD algorithm in 2017, which introduces a residual structure based on the SSD algorithm and uses ResNet-101 as the backbone network to form a “wide-narrow-wide” hourglass structure using deconvolution to fuse high-level semantic information with low-level semantic information, enriching the multiscale feature maps for predictive regression and classification detection tasks and improving the detection performance of small targets [32]. Due to the replacement of the backbone network, the number of parameters of the model increased sharply, which could not meet the needs of real-time detection. In 2018, Cui et al. and other researchers proposed the MD-SSD algorithm, which enhances the characteristics of small targets by introducing shallow and deep cross level connections and improves the detection accuracy of small targets [33]. MD-SSD simply fuses the shallow and deep feature layers to increase the information exchange between the feature layers and does not process the shallow feature layers to mine its own small target feature information. In 2020, researchers such as Zhai et al. proposed the DF-SSD algorithm, replacing the backbone network with DenseNet-S-32-1, which enhanced the feature extraction ability [34]. In 2021, researchers such as Chen and Luo proposed a method of integrating multiscale semantic information to enhance shallow features to detect small targets, which enhanced the detection effect of small targets and dense targets [35]. In reference 35, they perform a simple convolution process on the shallow feature layer, which loses a part of the required feature information during the convolution process and does not effectively extract the feature information of small targets. From the existing research results, on the basis of SSD detection algorithm, the feature information of the target to be measured is fused, which improves the robustness of the algorithm and improves the performance of small target detection. However, the existing research results do not effectively use the feature information contained in the shallow feature layer, resulting in the insufficient performance of the algorithm model in small target detection, and the detection accuracy still needs to be further improved.

In order to improve the detection performance and accuracy of the algorithm model for small targets, this paper proposes a MPH-SSD algorithm that combines the attention mechanism and multiscale double pyramid feature enhancement. First, the shallow feature enhancement module is designed to expand the receptive field of the shallow feature layer, enrich the semantic information in the feature layer for small targets, and enhance the expression ability of the shallow features. The multiscale information fusion module is used to select different scale feature layers for fusion, and the detail information in the shallow feature layer and the semantic information in the deep feature layer are fused. Secondly, the cascaded double pyramid structure is used to transfer from the deep layer to the shallow layer so that the context information between different feature layers can be effectively transferred, and the feature information can be further strengthened. The attention mechanism is used to enhance the feature response of the target to be detected and reduce the influence of the background on the detection performance of the algorithm.

## 2. Basic Model of the SSD Algorithm

An SSD algorithm is a single-stage target detection model based on regression. Using the idea of regression, the anchor box position and classification information of target information are directly regressed to the image. Using a priori frame mechanism, 4 ∼ 6 different numbers of default frames are extracted in each cell of the feature layer according to different length width ratio, and finally, 8732 default frames are obtained. The shallow feature map has rich spatial information and small receptive fields, which has a good effect on target positioning, but it lacks semantic information for classification, which has a poor effect on classification. On the contrary, the deep feature map has rich semantic information and large receptive fields, which can accurately classify targets. The shallow feature map has many pixels, which is suitable for small target detection, and the deep feature map has few pixels, which is suitable for large target detection [36].

The SSD algorithm takes VGG16 as its backbone network, replaces the last two layers of full connection with convolution layer network based on the original VGG16, uses the convolution layers with different convolution cores to extract more feature maps, and then extracts different size feature maps and VGG16 network feature maps from the convolution layer network to predict the detected targets independently. The structure of the SSD algorithm framework is shown in Figure 1. As you can see along the way, the algorithm resizes the input image to get a fixed size of 300 × 300 × 3 image, and the image is sent to the SSD network for processing, and then after the SSD feature extraction network, six different sizes of feature maps can be obtained, which are 38 × 38 × 512 of layer Conv4_3, 19 × 19 × 1024 of layer Fc7, 10 × 10 × 512 of layer Conv8_2, 5 × 5 × 256 of layer Conv9_2, 3 × 3 × 256 of layer Conv10_2, and 1 × 1 × 256 of layer Conv11_2. Feature extraction for targets of different scales is accomplished by different feature layers, in which the shallow feature layer mainly extracts feature information for small targets, and the deep feature layer mainly focuses on the feature information for large targets. Finally, the SSD algorithm sets a different number of priori anchors according to the aspect ratio of the size of the feature graph and obtains the boundary anchor of the object after processing by the nonmaximum suppression (NMS) algorithm.

## 3. Analysis of the MPH-SSD Algorithm Model

The traditional SSD algorithm detects targets by extracting different sizes of feature maps according to the algorithm itself, which can detect different targets. However, the shallow feature map lacks the semantic information of small targets, so the traditional SSD algorithm has insufficient performance in small target detection. To solve this problem, this paper presents an MPH-SSD optimization algorithm that combines the attention mechanism with multiscale double pyramid feature enhancement. The overall structure of the algorithm is shown in Figure 2.

From the diagram, it can be seen that there are four main modules in the algorithm, which are shallow feature enhanced module (SEM), multiscale feature fusion module (MFM), double pyramid feature enhancement module (DPEM), and hybrid attention module (HAM). This algorithm uses VGG16 as the backbone network and incorporates dilatation convolution to increase the perception field when the shallow features are extracted from the backbone network so as to obtain more and more abundant context information. At the same time, the deep feature layer is rich in semantic information, and the cascade multiscale double pyramid structure is used to enhance the deep feature layer and transfer the semantic information to the shallow feature layer. While transferring the semantic information from the deep feature layer to the shallow feature layer, it also ensures that the rich spatial information in the shallow feature layer can be transferred to the deep feature layer. Finally, the feature layer of different scales is used to fuse, and a multiscale information fusion module is constructed, which further fuses the semantic information and location spatial information to extract more context information, thus improving the detection effect of small targets.

### 3.1. Shallow Feature Enhanced Module

When processing feature information in the shallow feature layer, the semantic information of small targets is usually lost because of the small perceptual field. To solve this problem, a shallow feature enhancement module is designed to enable the algorithmic model to obtain a larger perceptual field and extract feature information at a higher semantic level. The structure of the shallow feature enhancement module is shown in Figure 3. The SEM designed in this paper has two main parts: the feature enhancement part and the connection part. The feature enhancement part is L2 to normalize the feature map to weaken the effect of large values of certain variables on the model and then perform three parallel expansion convolutions with expansion rates of 1, 2, and 3. First, the expansion convolutions with expansion coefficients of 1 and 2 are used to extract the spatial and location information of the small target, and then the expansion convolution with expansion rate of 3 is used to provide contextual information to the small target. Parallelizing the networks with three different sensory fields can effectively improve the continuity of features. The connection part preserves the feature information in the different inflated convolutional layers by the concatenate stacking operation. The concatenate operation is followed successively by a 3 × 3 convolution with the ReLu activation function and sigmoid activation function to adjust the size and the number of channels of the feature map. At the same time, a BN layer is added to speed up the training and convergence of the network to control the gradient explosion and to prevent overfitting. Finally, element-by-element multiplication is performed with the feature maps without any operation on the original input. The expansion convolutions of different expansion coefficients are connected together, which can effectively solve the problem of voids that exist after the convolution of different expansion coefficients, thus avoiding feature loss and improving the extraction performance of the shallow feature layer for small target features.

### 3.2. Multiscale Feature Fusion Module

In the SSD target detection algorithm, the feature information responsible for small target detection is mainly concentrated in the shallow feature layer. The shallow feature layer has higher resolution and richer detail information, but the shallow feature layer contains less semantic information, which leads to the general detection performance of small targets.

To solve this problem, this paper designs a multiscale feature fusion module, whose structure is shown in Figure 4.

In MFM, three feature layers with different depths and scales are selected for fusion. The purpose is to fuse the location and spatial information contained in the shallow feature layer with the semantic information in the deep feature layer so as to improve the detection performance of this algorithm MPH-SSD for small targets. The principle of multiscale feature fusion is

(1) $$\begin{array}{c} X_{f}=\phi_{f}\left\{T_{1}\left(X_{1}\right),T_{2}\left(X_{2}\right),T_{3}\left(X_{3}\right)\right\}\text{.} \end{array}$$

Among them, *X*_1_, *X*_2_, and *X*_3_ represent the feature layer that needs feature fusion in VGG16 feature extraction network; *T*_1_, *T*_2_, and *T*_3_ represent the transformation that needs to be carried out before the feature layer is fused; and the feature layers of different scales that need to be fused are transformed to the same scale for stacking fusion. The subscript *f* represents the feature fusion function. In the multiscale information fusion module designed in this paper, the concatenate operation is adopted. *X*_*f*_ is the fusion features obtained after the fusion operation. The process of feature fusion is such that the third and fourth layers processed by the shallow feature enhancement module and the ninth feature layer extracted by the VGG16 backbone network are used as the input of the multiscale fusion module. First, layer Conv3_3 and layer Conv4_3 use 3×3 convolution scales to 64 × 64 × 512, and then layer Conv9_1 feature layer uses 1 × 1 deconvolution scales to 64 × 64 × 512. Finally, concatenate stacking is used to join the three different scales of feature layers to fuse the rich detail information in the shallow feature layer and the rich semantic information in the deep feature layer into a feature map. After fusing layer Conv4_3, layer Fc7, layer Conv10_1 and layer Conv5_3, and layer Conv8_2 and layer Conv11_1, we can get the fuse features of Fuse1, Fuse2, and Fuse3 at different scales.

### 3.3. Double Pyramid Feature Enhancement Module

Feature pyramid is a top-down structure for multiscale fusion of feature information, which can solve the problem that it is difficult to deal with multiscale features in the process of target detection. Because the feature pyramid is one-way transmission of feature information, it is easy to lose some detail feature information in the process of feature enhancement. Therefore, the effect of feature pyramid on the improvement of algorithm model is limited [37].

To solve this problem, a double pyramid feature enhancement module is designed, and its structure is shown in Figure 5(a). From the figure, it can be seen that on the basis of the original pyramid structure, a channel that can be directly connected to the output is added, which is similar to the network structure of jump connection in U-Net network [38]. Before DPEM, the deep features extracted by VGG16 are enhanced, and the context information in the deep feature layer of different scales is extracted in parallel, and they are fused with the semantic information in the deep feature layer. The three fusion features and enhanced deep features generated in the multiscale fusion module are used as the input of DPEM. The addition of ECA (Efficient Channel Attention) makes the deep features more focused on capturing cross-channel interaction information, avoiding the deep network from missing information due to dimensionality reduction. The structure is shown in Figure 5(b). Different from the traditional pyramid structure, the double pyramid structure designed in this paper adds a bottom-up feature transmission channel on the original basis and adds a channel between the same nodes that can be directly connected to the output, which enriches the feature information and makes the feature information in the network structure more accurately expressed.

### 3.4. Hybrid Attention Module

Since the feature maps have different scales and different perceptual fields, there are differences between feature information, and the use of common feature fusion methods does not effectively reflect the correlation and importance of channel and spatial features in features of different scales, which will produce overlap effects and position shifts in the target detection process and eventually brings negative impacts to the target detection task. To address this problem, the hybrid attention mechanism module structure designed in this paper is shown in Figure 6, with the upper part performing channel attention and the lower part performing spatial attention [39]. The CBAM attention mechanism is changed from the original serial connection to parallel fusion to form an improved CBAM attention mechanism module, which focuses not only on the correlation between channels but also on the relationship of feature information in terms of location, which helps the network to detect the target more accurately.

To further focus on the location information of the target in the detection image, the improved CBAM attention mechanism module in this paper is followed by a tandem fusion of the location attention module. The rich location information in the shallow feature map is used to extract the dependency between two random locations in the feature map, and for the feature information at a specific location, it will be weighted by all the feature information at that location and updated for that location. The weight is the similarity between the corresponding two positions, so this makes any two positions with similar features optimize each other, while ignoring the distance between these two positions. The impact of the background and the negative information generated during feature fusion is reduced, more contextual information is retained in the network, attention is preferentially allocated to key feature information that is more valuable for the target detection task, and the feature map after summation fusion can be adaptively adjusted.

The channel features *E*_*i*_ and spatial features *S*_*i*_ are obtained by the channel attention module and spatial attention mechanism, respectively, and then the two feature maps are summed element-by-element to generate the feature map *D*_*i*_. After three parallel 1 × 1 convolutions with the ReLU activation function, three feature maps *D*_*i*1_, *D*_*i*2_, and *D*_*i*3_ are generated; subsequently, the feature map *D*_*i*1_ is converted into an *N* × *C* matrix *D*_*i*1_^*T*^ by reshape operation and transpose operation, and the feature map *D*_*i*2_ is converted into a *C* × *N* matrix *D*_*i*2_′ by transpose operation, where *N*=*W*×*H*; then the matrix *D*_*i*1_^*T*^ and the matrix *D*_*i*2_′ are subjected to matrix product operation to obtain the correlation matrix *R*, the process of which can be expressed as follows:

(2) $$\begin{array}{c} \left\{\begin{array}{c} D_{i}=E_{i}+S_{i}\text{,}\\ D_{i1}=\text{Conv}\left(D_{i}\right)\text{,}\\ D_{i2}=\text{Conv}\left(D_{i}\right)\text{,}\\ D_{i3}=Conv\left(D_{i}\right)\text{,}\\ D_{i1}^{T}=Tran\left(Re\left(D_{i1}\right)\right)\text{,}\\ D_{i2}^{\prime }=Tran\left(D_{i2}\right)\text{,}\\ R=D_{i1}^{\prime }\cdot D_{i2}^{\prime }\text{.} \end{array}\right. \end{array}$$

In formula (2), Conv() denotes the 1 × 1 convolution function with the ReLU activation layer, Tran() denotes the transpose function, and Re() denotes the reshape function. After obtaining the correlation matrix *R*, it is necessary to perform reshape operation on *R* to convert *R* into feature map *R*^*R*^, and then it is necessary to perform average pooling and sigmoid activation operation on *R*^*R*^ to obtain the attention matrix *A*. Finally, the attention matrix *A* and the feature map *D*_*i*3_ are multiplied element-by-element and then added with the feature map *D*_*i*_ element-by-element to obtain the final feature map containing the detection target location information *P*_*i*_, then the process can be expressed as

(3) $$\begin{array}{c} \left\{\begin{array}{c} R^{R}=Re\left(R\right)\text{,}\\ A=\phi \left(\text{Avg}\left(R^{R}\right)\right)\text{,}\\ P_{i}=A⊗D_{i3}⊕D_{i}\text{.} \end{array}\right. \end{array}$$

In formula (3), ⊕ denotes element-by-element summation, and *P*_*i*_ is used as the output of the location attention module and also as the input of the prediction layer of the model in this paper. The hybrid attention module can enhance the representation of the feature layer at key locations and highlight the importance of the target location.

## 4. Experiments and Analysis of Results

### 4.1. Experimental Set-Up

In order to verify the effectiveness of the design method, two datasets, VOC07 + 12 (PASCAL VOC2007 plus PASCAL VOC2012) and MS COCO, were used to validate the algorithm. The PASCAL VOC dataset is a standardized dataset provided by the official PASCAL VOC Challenge. The VOC07 + 12 dataset contains 20 categories (plus background for a total of 21 classifications), which contains 16,551 training images for a total of 40,058 targets, 8,333 validation images for a total of 20,148 targets, and 4,952 test images for a total of 12,032 targets. The MS COCO dataset selected in this experiment is COCO2017, which is divided into 80 object categories in the target detection task, and the dataset contains 118,287 training images, 5,000 validation images, and 40,670 test images, in which the majority of targets are from real-life example images, with rich target scenes and a large number of small target objects, which are suitable for the performance evaluation of target detection algorithms.

The model of the optimization algorithm in this paper is based on the TensorFlow 2.0 framework with Python version 3.7. The experimental environment used in the training experiments is NVIDIA Tesla V100s 32GB GPU, and the weights of the backbone network are obtained by pretraining on ImageNet. The SGD (stochastic gradient descent) algorithm was used in the experiments, and the initial learning rate was set to 0.002. Cosine annealing was used to adjust the learning rate of the model during the training process, and the momentum was set to 0.937. To prevent overfitting and promote convergence, the decay weight was set to 0.0005. In the experimental process, two images with different sizes are used as the input of the algorithm model in this paper. When the input image size is 300 × 300, the batch_size of the model is set to 32, and when the input image size is 512 × 512, the batch_size of the model is set to 16.  Figure 7 shows the training loss profile of the MPH-SSD model. As can be seen in Figure 7(a), the loss value decreases rapidly from 17 on the VOC dataset and finally converges around 3.5, and from Figure 7(b), it can be seen that the loss value decreases rapidly from 25 on the COCO dataset and finally converges around 4, indicating that the model achieves good results after sufficient training. When MPH-SSD was trained on the VOC dataset, the learning rate decreased by a factor of 10 after the completion of the 125th and 175th iterations, respectively, and the whole experiment converged after the completion of the 196th iteration to obtain the final network model weights. When the training experiments were performed on the COCO2017 dataset, the learning rate was decreased by a factor of 10 after the completion of the 200th and 250th iterations, respectively, and the whole experiment converged after the completion of the 292th iteration to obtain the final network model weights.

### 4.2. Analysis of Results

In order to verify whether the algorithm of this paper is effective, in this section, we mainly compare the performance of the proposed SSD optimization algorithm MPH-SSD, which integrates the attention mechanism and multiscale double pyramidal feature enhancement, with the target detection algorithm based on CNN in recent years, and we can see from the comparison results that the target detection algorithm proposed in this paper has better performance in small target detection.

#### 4.2.1. Performance Comparison on the PASCAL VOC Dataset

Table 1 lists the experimental results comparing the algorithms in this paper and recent years' convolutional neural network-based target detection algorithms on the PASCAL VOC dataset. The experimental results of these algorithms were obtained using the training and validation sets of both VOC2007 and VOC2012 as training sets. The mAP (mean Average Precision) in Table 1 is the average of the average precision values of each category detected with a positive and negative sample region intersection ratio of 0.5. Fps indicates the number of images that the algorithm can process per second, which is not only related to the algorithm model but also the hardware configuration of the experiment.

From the results listed in Table 1, we can see that the MPH-SSD algorithm proposed in this paper achieves 82.1% detection accuracy and 53.5 frames detection speed when the input image size is 300 × 300, and 87.7% detection accuracy and 24.6 frames detection speed when the input image size is 512 × 512, which ensures real-time detection speed while maintaining a high detection accuracy. The MPH-SSD algorithm in this paper also shows a 1.6% improvement in detection accuracy compared to the RFB algorithm for an input size of 300 × 300, a 4.9% improvement in detection accuracy compared to the classical SSD algorithm, and a 3.5%, 3.5%, 3.2%, 2.5%, 3.6%, and 3.3% improvement compared to the improved family of SSD-based DSSD, MD-SSD, DF-SSD, SEFN, RSSD, and FSSD algorithms, respectively, and 3.5%, 3.2%, 2.5%, 3.6%, 3.3% and 28.8%, 12.15%, and 8.9% improvement in detection accuracy compared to several classical two-stage target detection (R-CNN, Fast R-CNN, and Faster R-CNN), respectively. There are also 18.7%, 8.4%, and 2.5% improvements in detection accuracy compared to the more popular one-stage algorithms YOLOv1, YOLOv2, and YOLOv3. There is a 5.5% improvement compared to the RFB algorithm in the case of 512 × 512 input size, 9.2% improvement in detection accuracy compared to the classical SSD algorithm, 6.2%, 6.7%, 6.5%, 6.9%, and 6.8% improvement compared to DSSD, MD-SSD, SEFN, RSSD, and FSSD algorithms based on the improved series of SSD, and several classical two-stage target detection methods (R-CNN, fast R-CNN, and faster R-CNN) improved the detection accuracy by 34.4%, 17.7%, and 14.5%, respectively. Compared to the more popular one-stage algorithms YOLOv1, YOLOv2, and YOLOv3, there is a 24.3%, 14%, and 9.1% improvement in detection accuracy, respectively.

Figure 8 shows the detection accuracy of the algorithm in this paper and several SSD-based optimization algorithms, namely SSD, DF-SSD, DSSD, and RSSD, for 20 classifications on the PASCAL VOC dataset. From Figure 8, it can be seen that the detection accuracy of this paper's algorithm MPH-SSD in these 20 categories has been greatly improved in all categories except for the slight shortage of detection accuracy in individual classes, especially in the small target classification, where the performance improvement is particularly obvious.

Different network construction methods have different accuracy and speed. To better demonstrate the trade-off between accuracy and speed of the algorithm in this paper, Figure 9 shows the comparison between the algorithm in this paper and other algorithms in these two metrics. Figure 9(a) shows map-fps performance for small input sizes, and Figure 9(b) shows map-fps performance for large input sizes. From the figure, it can be seen that the MPH-SSD algorithm in this paper can strike a good balance between accuracy and speed without giving up one metric at the expense of the other in the excessive pursuit of one metric, no matter in the case of small-size input or large-size input.

Table 2 lists the test results of different types of algorithms on the VOC07 + 12 dataset for the four small target categories such as boat, chair, plant, and bottle. From the experimental results with an input size of 300 × 300, it can be seen that the detection performance of the proposed algorithm MPH-SSD in this paper for small target classification in the VOC dataset is more significantly improved compared with other algorithms.

To verify the effectiveness of the MPH-SSD algorithm on small target detection, this paper conducts ablation experiments on the VOC 07 + 12 dataset by gradually adding a shallow feature enhancement module (SEM), a multiscale feature fusion module (MFM), a double pyramid feature enhancement module (DPEM), and a hybrid attention module (HAM) to the basic SSD model and by comparing the detection accuracy differences to analyze the performance of each module of the MPH-SSD algorithm. The results of the ablation experiments are shown in Table 3.

In order to verify the effectiveness of SEM, the ablation experiment is based on the traditional SSD algorithm, and SEM is added to the shallow feature layer part to enhance the shallow features to improve the model's perception of small target features. The mAP of the model is improved by 2.8% compared with the SSD algorithm, which proves that SEM can provide more feature information to the model and is beneficial to the small target detection performance.

To verify the effectiveness of MFM, the ablation experiment adds three MFM modules to the traditional SSD algorithm and fuses feature maps at different scales through concatenate operation. After adding MFM, the model mAP is improved by 4.2% compared with the SSD algorithm, which proves that MFM can provide help for the model to fuse location space information and semantic information in different feature layers.

To verify the effectiveness of DPEM, the ablation experiment added DPEM to SEM and MFM, and the mAP of the model improved by 3.8%, proving that DPEM can provide the model with contextual information at different scales and enable more accurate representation of feature information in the network structure.

To verify the effectiveness of HAM, the ablation experiment added HAM to the first three modules, and the mAP of the model improved by 1.7%, proving that HAM contributed to reducing the background as well as the impact of negative information generated in the feature fusion process, alleviating the problem of information imbalance between feature maps in the feature fusion process.

#### 4.2.2. Comparison of the Actual Detection Effect of Different Detection Methods

Figure 10 shows the comparison of the image detection effect of this paper's algorithm MPH-SSD with the classical SSD algorithm and DSSD algorithm on the PASCAL VOC dataset. From the comparison results in Figure 10, it can be concluded that the SSD algorithm is obviously insufficient for the detection of small targets and often has the phenomenon of missed detection. Although the DSSD algorithm is optimized on the basis of the SSD algorithm, which improves the situation of missed detection of targets by the SSD algorithm, there is the situation of missed detection of small targets and clustered targets in the detection of small targets. In contrast, the SSD optimization algorithm that incorporates the attention mechanism and multiscale double pyramidal feature enhancement used in this paper can effectively improve the detection performance of small targets, which is especially effective in the case of large-size image input.

#### 4.2.3. Performance Comparison on the MS COCO Dataset

To further illustrate the performance advantage of this paper's algorithm for small target detection, it was also tested on the MS COCO dataset, and the results were also compared with other methods from the literature, as shown in Table 4, where “iou = 0.5:0.95” means that 10 thresholds are set in steps of 0.05 between 0.5 and 0.95, and the average accuracy corresponding to each threshold is taken as the average, where “S, M, L” means small target, medium target, and large target, respectively. From the results in Table 4, it can be seen that this method has significantly improved the detection accuracy and recall rate compared with Faster R-CNN, Mask R-CNN, YOLOv2, SSD512, DSSD513, DF-SSD, SEFN512, FSSD512, and RFB512. The results in Table 4 effectively prove that the algorithm in this paper has good performance in small target detection.

## 5. Conclusion

In order to improve the detection performance of small targets during target detection, an MPH-SSD optimization algorithm that fuses the attention mechanism and multiscale double pyramid feature enhancement is proposed in this paper. Based on the SSD algorithm, four modules are designed: shallow feature enhancement module, multiscale feature fusion module, dual pyramid feature enhancement module, and hybrid attention module. First, we increase the perceptual field of the shallow feature layer to enrich the semantic information of the shallow feature layer by expanding the convolution and make the regions containing small targets in the shallow feature layer enhanced by the original spatial information and semantic information. Then, the enhanced feature map is fused with the deep feature layer to improve the semantic information of the shallow feature layer and the detail information of the deep feature layer while also improving the feature extraction and feature generalization ability of the model. Then, a double pyramid structure is used to construct a bottom-to-top feature transmission channel to enrich the feature information to further enhance the feature information of small targets. Finally, a hybrid attention mechanism is used to retain more contextual information in the network, adaptively adjusting the feature maps after summation and fusion to reduce background interference. The MPH-SSD algorithm is experimentally analyzed on PASCAL VOC and MS COCO datasets, and the mAP of this paper's algorithm is 87.7% and 51.1%, respectively. The results show that the MPH-SSD algorithm can better utilize the feature information in the shallow feature layer in the small target detection process and has better detection performance for small targets. Although the algorithm in this paper achieves improvement in small target detection accuracy, the dual-feature pyramid enhancement module increases the network computation to a certain extent, which makes the algorithm speed down slightly. How to reduce the redundancy and optimize the network structure while ensuring the accuracy will be the main direction of future research.

## Figures and Tables

**Figure 1:** SSD algorithm framework diagram.

**Figure 2:** MPH-SSD algorithm network structure.

**Figure 3:** Shallow feature enhanced module structure diagram.

**Figure 4:** Multiscale feature fusion module structure diagram.

**Figure 5:** Double pyramid feature enhancement module and ECA module. (a) Double pyramid feature enhancement module structure diagram. (b) ECA module.

**Figure 6:** Hybrid attention mechanism module structure diagram.

**Figure 7:** MPH-SSD model training loss curve. (a) Training loss curve of the PASCAL VOC dataset. (b) Training loss curve of the COCO dataset.

**Figure 8:** Comparison of detection accuracy between the MPH-SSD algorithm and other algorithms in PASCAL VOC dataset 20 classification.

**Figure 9:** The mAP-FPS plots of the algorithm in this paper and other algorithms. (a) mAP-FPS plots of small-size input. (b) mAP-FPS plots of large-size input.

**Figure 10:** Comparison of detection effects of different algorithms on the PASCAL VOC dataset.

**Table 1:** Performance comparison of the MPH-SSD algorithm and other algorithms on the PASCAL VOC dataset.

Methods	Backbone	Size	mAP (%)	Fps
R-CNN [25]	AlexNet	227 × 227	53.3	—
Fast R-CNN [27]	VGG16	224 × 224	70.0	—
Faster R-CNN [28]	VGG16	1000 × 600	73.2	7.0
Faster R-CNN [28]	ResNet-101	1000 × 600	76.4	2.4
YOLOv1 [30]	GoogleNet	448 × 448	63.4	45.0
SSD300 [31]	VGG16	300 × 300	77.2	46.0
SSD512 [31]	VGG16	512 × 512	78.5	19.0
DSSD321 [32]	ResNet-101	321 × 321	78.6	9.5
DSSD513 [32]	ResNet-101	513 × 513	81.5	5.5
MDSSD300 [33]	VGG16	300 × 300	78.6	32.2
MDSSD512 [33]	VGG16	512 × 512	81.0	14.5
DF-SSD [34]	DenseNet-S-32-1	300 × 300	78.9	11.6
SEFN300 [35]	VGG16	300 × 300	79.6	55.0
SEFN512 [35]	VGG16	512 × 512	81.2	30.0
YOLOv2 [40]	Darknet19	352 × 352	73.7	81.0
YOLOv3 [41]	Darknet19	320 × 320	79.6	52.2
RSSD300 [42]	VGG16	300 × 300	78.5	35.0
RSSD512 [42]	VGG16	512 × 512	80.8	16.6
FSSD300 [43]	VGG16	300 × 300	78.8	65.8
FSSD512 [43]	VGG16	512 × 512	80.9	35.7
RFB300 [44]	VGG16	300 × 300	80.5	83.0
RFB512 [44]	VGG16	512 × 512	82.2	38.0
MPH-SSD300	VGG16	300 × 300	82.1	53.5
MPH-SSD512	VGG16	512 × 512	87.7	24.6

**Table 2:** Comparison of detection performance of different algorithms on the small target classes of PASCAL VOC dataset.

Methods	mAP (%)	Boat	Chair	Plant	Bottle
R-CNN [43]	53.3	36.8	27.9	29.5	35.9
Fast R-CNN [36]	70.0	52.3	44.2	35.1	38.7
SSD [40]	77.2	61.9	58.1	50.2	47.6
DSSD [41]	78.6	64.6	59.5	53.3	46.8
DF-SSD [43]	78.9	65.8	62.4	51.9	51.3
FSSD [42]	78.8	72.3	66.8	56.9	59.7
MPH-SSD	82.1	75.4	67.1	64.3	62.4

**Table 3:** Analysis of ablation experiment results.

SEM	MFM	DPEM	HAM	VOC 07 + 12
				mAP (%)
				72.4
√				75.2
√	√			76.6
√	√	√		80.4
√	√	√	√	82.1

**Table 4:** Performance comparison of the MPH-SSD algorithm and other algorithms on the MS COCO dataset.

Method	Backbone network	Avg. precision, IoU			Avg. precision, area			Avg. recall, area		
		IoU = 0.5 : 0.95	IoU = 0.5	IoU = 0.75	Area : S	Area : M	Area : L	Area : S	Area : M	Area : L
Faster R-CNN [37]	VGG16	24.2	45.3	23.5	7.7	26.4	37.1	—	—	—
Mask R-CNN [29]	ResNeXt-101-FPN	37.1	60.0	39.4	16.9	39.9	53.5	—	—	—
YOLOv2 [40]	Darknet19	21.6	44.0	19.2	5.0	22.4	35.5	9.8	36.5	54.4
SSD512 [40]	VGG16	27.7	46.4	26.7	10.9	31.8	43.5	16.5	46.6	60.8
DSSD513 [41]	ResNet-101	33.2	53.3	35.2	13.0	35.4	51.1	28.9	43.5	46.2
DF-SSD [43]	DenseNet-S-32-1	29.5	50.7	31.3	9.8	31.1	46.5	17.3	46.8	64.4
SEFN512 [44]	VGG16	33.7	54.7	35.6	19.2	38.0	47.3	29.1	52.5	63.2
FSSD512 [43]	VGG16	31.8	52.8	33.5	14.2	35.1	45.0	22.3	49.9	62.0
RFB512 [44]	VGG16	34.4	55.7	36.4	17.6	37.0	47.6	27.3	52.3	65.4
MPH-SSD	VGG16	51.1	79.8	55.6	21.1	36.3	59.4	28.4	46.8	67.9

## Data Availability

The data used to support the findings of this study are available from the corresponding author upon request.
